# Targetting an LncRNA P5848-ENO1 axis inhibits tumor growth in hepatocellular carcinoma

This article has been retracted.

**DOI:** 10.1042/BSR20180896

**Published:** 2019-11-15

**Authors:** Xidan Zhu, Hui Yu, Baolin Li, Jing Quan, Zhangrui Zeng, Guangrong Li, Jinbo Liu

**Affiliations:** Department of Laboratory Medicine, The Affiliated Hospital of Southwest Medical University, Luzhou 646000, Sichuan, China

**Keywords:** Hepatocellular carcinoma (HCC), LncRNA P5848, ENO1, Therapeutic target

## Abstract

Hepatocellular carcinoma (HCC) has a high recurrence rate and poor clinical outcome after currently used therapies, including radiofrequency ablation. To explore the possible mechanisms for the relapse of HCC, in the present study we focussed on long non-coding RNA (LncRNA), which has been reported to be involved in tumorigenesis. We identified an LncRNA P5848, whose expression level was up-regulated in tumor samples from HCC patients after radiofrequency ablation. As such, we speculated that LncRNA P5848 may play a role in tumor growth. Here we showed that LncRNA P5848, whose up-regulation can lead to HCC cancer cell proliferation and migration. *In vitro* and *in vivo* overexpression of LncRNA P5848 promoted cell growth, cell survival, and cell invasion, whereas LncRNA P5848 depletion exerts opposite effects. Mechanistically, we have found that ENO1 was the target of LncRNA P5848. LncRNA P5848 up-regulated the gene and protein expression level of ENO1, promoting tumor growth and cell survival. However, siRNA-mediated knockdown of ENO1 counteracted the effects of LncRNA P5848 on cancer cell growth, cell survival, and migration. Taken together, LncRNA P5848 promotes HCC development by up-regulating ENO1, indicating that LncRNA P5848-ENO1 axis is a potential therapeutic target for the treatment of HCC.

## Introduction

Hepatocellular carcinoma (HCC) is a common and deadly cancer, constituting the second most common cause of cancer deaths in developing nations and the sixth most common cause in developed countries [1]. Despite considerable efforts and advances aimed at understanding HCC-related tumorigenesis, metastasis, and treatment, morbidity and mortality continue to rise [2]. One driver of HCC mortality is that most patients have advanced disease at diagnosis, often systemic metastases. A detailed understanding of the mechanisms of HCC metastasis is required to identify innovative therapeutic options.

Radiofrequency ablation is a currently used therapeutic strategy for the treatment of HCC in the clinic, however, the relapse often occurs, which acquires the mechanistic exploration. Accumulating evidence suggests that long non-coding RNA (LncRNA) has been implicated in the tumorigenesis via regulating cancer cell proliferation, cell survival, and migration/metastases [3,4]. Of note, epithelial to mesenchymal transition (EMT) plays a pivotal role in the development of cancerous metastases wherein tumor cells acquire migratory characteristics, often dependent on a reduction in the expression of cell adhesion molecules [5]. Prior studies have established the link between EMT processes and signaling pathways associated with drug resistance and tumor relapse [6–8]. Thus, exploration of the role of LncRNA in tumorigenesis will provide new clues for further understanding the molecular mechanisms. The tumor hyperthermia has been listed as the sixth anticancer strategy after surgery, radiotherapy, chemotherapy, targetted therapy, and immunotherapy. It has many advantages, being non-invasive, painless, safe and reliable and easy to operate. Our previous experiment showed that LncRNA P5848 was up-regulated after heat exposure and combined with hyperthermia for tumor killing.

In the present study, we studied the role of LncRNA P5848 in HCC *in vitro* and *in vivo*, with a focus on the effects on cell proliferation, apoptosis, and migration. Also, we investigated the molecular target of LncRNA P5848 to explain the role of LncRNA P5848 in HCC. At last, we examined the antitumor effect via targetting LncRNA P5848-ENO1 axis for the treatment of HCC *in vivo*. In addition to these mechanisms, discovery of additional pathways involved in HCC development and progression may lead to new therapeutic opportunities. We preliminarily speculate LncRNA P5848 could be an explanation for HCC relapse and function as a potential target for HCC therapy.

## Materials and methods

### Cell culture

Liver cancer cell lines HepG2, SMMC-7721, and MHCC97-H, were purchased from Cell Bank of Typical Culture Preservation Committee of Chinese Academy of Science (Shanghai, China). Cell lines were cultured in DMEM medium (Invitrogen, Carlsbad, CA, U.S.A.) supplemented with 10% FBS (HyClone, Logan, UT, U.S.A.) in a humidified atmosphere of 5% CO_2_ at 37°C.

### Heat treatment

#### Quantitative real-time PCR

Quantitative real-time PCR (qRT-PCR) assays were performed as previously described [9]. Briefly, total RNA was isolated by TRIzol Reagent (Life Technologies, Carlsbad, CA) from the frozen tissue samples or HCC cell lines according to the manufacturer’s protocol. cDNA was obtained from RNA using a universal cDNA synthesis kit (TAKARA, Shiga, Japan). Resultant products were amplified using a SYBR Green PCR kit (Toyobo, Tokyo, Japan) for qRT-PCR analysis. Amplification plots were analyzed by Bio-Rad IQ5 software (Bio-Rad Laboratories Inc, California, U.S.A.). All quantitations were normalized to the level of endogenous GAPDH as a control [9]. All primers were purchased from GeneCopia (Rockville, MD, U.S.A.).

#### Western blot analysis

Cell lysate was fractionated by SDS/PAGE, then transferred to PVDF membrane (Roche Life Sciences, Switzerland). Membranes were blocked with 5% skim milk in TBST for 1 h at room temperature, then incubated with primary antibody overnight at 4°C. β-actin was used as a loading control. After incubation, the membranes were washed by TBST and incubated with HRP–conjugated secondary antibody, and the antigen–antibody complex was detected with ECL reagents (Meck Millipore, Massachusetts, U.S.A.). Antibodies are listed in the Supplementary Table S1.

### *In situ* hybridization protocol

Fluorescence *in situ* hybridization (FISH)—P5848 RNA probes were synthesized and labeled with Alexa Fluor 594 using the FISH Tag RNA Multicolor kit (Life Technologies, Gaithersburg, MD). Cells grown on cover glasses were treated with 20 µg/ml proteinase K at 37°C for 1 h and washed with 2× SSC solution followed by water at room temperature. The cells were then incubated with pre-denatured P5848 probes in a dark and humid environment at 55°C for 24 h to allow hybridization. The cells were then washed with 50% formamide in 2× SSC for four times before P5848 in SMC differentiation mounting. Nuclei were counterstained with 5,6- DAPI.

### Luciferase activity assay

Luciferase reporter assay—250 ng of either empty vector or p5848 was co-transfected with 250 ng of firefly luciferase reporter driven by ENO1 promoter into 293T cells in 12-well plates using Lipofectamine LTX (Invitrogen, U.S.A.). Then luciferase activities were measured using a luciferase assay kit (Promega) according to the manufacturer’s protocol. The experiments were repeated for three times with triplicates.

### Immunofluorescence

Cells were seeded on coverslips, then fixed with 4% paraformaldehyde in PBS for 15 min, and washed twice with PBS. Primary antibodies against E-cadherin (Proteintech Group, Chicago, U.S.A.) and N-cadherin (Cell Signaling Technology) were incubated overnight at 4°C. ENO1 was visualized using FITC–conjugated goat anti-mouse or anti-rabbit IgG (Genecopia, Guangzhou, China). DAPI was used as a nuclear counter stain (Genecopia, Guangzhou, China). Leica DMRA fluorescence microscope (Leica, Wetzlar, Germany) was used to obtain the images.

### MTT assay

Cell growth was examined using MTT assays.

### Migration assay

Cell migration and invasion were tested using Transwell assay plates (Corning, New York, U.S.A.). Cells were placed into the upper chamber of the insert with matrigel (Corning, New York, U.S.A.). After 48 h incubation at 37°C, cells adhering to the lower membrane of the insert were stained with 0.1% Crystal Violet and counted using a Leica microscope (Leica, Wetzlar, Germany).

### Animal experiments

All experimental procedures involving animals were in accordance with the Guide for the Care and Use of Laboratory Animals (NIH publication no. 80-23, revised 1996) and were performed according to the institutional ethical guidelines for animal experiments. All studies involving animals were approved by the Affiliated Hospital of Southwest Medical University. Male BALB/C nude mice (5 weeks old) were raised under SPF environment in the animal facility during the experiment procedures with free access to diet or water. Briefly, 4 × 10^6^ cells in 100 µl PBS were injected subcutaneously into the flanks of nude mice. After 6 weeks, the subcutaneous tumors were resected and cut into 1 mm^3^ pieces, then implanted into left liver to mimic primary HCC. Ten animals were randomly divided into each study group. Eight weeks after implantation, mice were killed and the livers were analyzed by standard histological examination.

### Statistical analysis

Statistical analyses were performed by SPSS 17.0. Data was expressed as the mean ± S.E.M. from at least three independent experiments. Quantitative data were compared between groups using the Student’s *t* test. *P*-values of less than 0.05 were considered significant.

## Results

### LncRNA P5848 was up-regulated after heat exposure

Since there are compelling evidence showing that LncRNAs have been implicated in tumor onset, progression, and metastasis, in the present study we focussed on the role of LncRNA in HCC. To start the study on the role of LncRNA P5848 in HCC, we first noticed the relapse of HCC after radiofrequency ablation in patients in the clinic and we found that the expression of LncRNA P5848 was increased after heat and radiofrequency ablation via Chip data (Figure 1A,B). Following this intriguing finding, we tested the expression level of LncRNA P5848 in three different HCC cell lines. To mimic the condition of radiofrequency ablation, cells were exposed to heat at 50°C. The expression level of LncRNA P5848 was increased in SMMC-7721, MHCC97-H, and HepG2 cells after exposure to 50°C, and the level of LncRNA P5848 was significantly increased after 48 h (Figure 1C–E). Apart from that, the subcellular distribution of LncRNA P5848 in HCC cell lines was examined. As shown in Figure 1F, LncRNA P5848 transcripts were detected by *in situ* hybridization of Cy3-tagged oligonucleotides that hybridize to the hairpin ribozyme insert (red). The location of nuclei is indicated by Hoechst staining (blue). Thusly, taken together, the initial data show that heat shock induces the expression of LncRNA P5848, which could be an explanation for HCC relapse and functions as a potential target for HCC therapy.

**Figure 1:** Expression level of LncRNA P5848 (**A**) The heat map for the expression of lncRNA when treated with heat. (**B**) The expression level of LncRNA P5848 was up-regulated in HCC tumor after radiofrequency ablation. The expression level of LncRNA P5848 was increased after heat exposure for 48 h (**C**); the level of LncRNA P5848 was increased in SMMC-7721, MHCC97-H, and HepG2 cells after exposure to 50°C (**D,E**). (**F**) Subcellular distribution of LncRNA P5848 in HCC cells. LncRNA P5848 transcripts were detected in HepG2, MHCC97-H, and SMMC-772 by *in situ* hybridization of Cy3-tagged oligonucleotides that hybridize to the hairpin ribozyme insert (red). The location of nuclei is indicated by Hoechst staining (blue). *P<0.05, **P<0.01.

### Effects of LncRNA P5848 on cell proliferation, apoptosis, and migration

After we observed the increase in LncRNA P5848 expression upon the heat exposure, we carried out experiments to test our hypothesis that LncRNA P5848 promotes HCC tumor growth. We examined the effect of LncRNA P5848 on cell growth, apoptosis, and migration (Figure 2). We found that LncRNA P5848 promoted cell growth, inhibited cell apoptosis; whereas knockdown of LncRNA P5848 induced apoptosis (Figure 2A,B). We also tested the activation of caspase cascade. Knockdown of LncRNA P5848 increased the expression level of pro-apoptotic protein BAX and induces caspase-3 cleavage, while decreasing the level of anti-apoptotic protein Bcl-2 (Figure 2C). In addition, LncRNA P5848 promoted cell migration, while knockdown of LncRNA P5848 inhibited cell migration (Figure 2D). In aggregates, the data suggest that LncRNA P5848 promotes tumor cell growth and survival.

**Figure 2:** Effects of LncRNA P5848 on cell proliferation, apoptosis, and migration (**A**) LncRNA P5848 promotes cell growth. HepG2 were heated at 50°C over 72 h, resulting in a remarkable increase in cell growth compared with other treatments. (**B**) LncRNA P5848 inhibits cell apoptosis, whereas knockdown of LncRNA P5848 induces apoptosis. (**C**) Representative blots showing the expression level of BAX, Bcl-2, Cleaved caspase-3. β-actin functions as an internal loading control. Heat exposure increases anti-apoptotic protein Bcl-2, while decreasing BAX. Knockdown of LncRNA P5848 increases the expression level of pro-apoptotic protein BAX and induces caspase-3 cleavage, while decreasing the level of anti-apoptotic protein Bcl-2. (**D**) LncRNA P5848 promotes cell migration, while knockdown of LncRNA P5848 inhibiting cell migration. *P<0.05, **P<0.01.

### LncRNA P5848 inhibits ENO1 expression

To further explain the cell growth promoting effect of LncRNA P5848 on tumor growth, we explored the molecular target of LncRNA P5848. We found that LncRNA P5848 promoted ENO1 expression, whereas knockdown of LncRNA P5848 suppressed ENO1 expression (Figure 3A). LncRNA P5848 also enhanced *ENO1* mRNA expression, while knockdown of LncRNA P5848 decreased *ENO1* mRNA expression (Figure 3B). To further confirm the targetting effect of LncRNA P5848 on ENO1, we carried out a luciferase assay as presented in Figure 3C, the data showed that heat exposure significantly increased luciferase activity, whereas knockdown of LncRNA P5848 markedly reduced the activity which was similar to the effect of ENO1 knockdown (Figure 3D), indicating that LncRNA P5848 targets ENO1. Furthermore, the immune-fluorescence assay also showed an increase in ENO1 expression in the presence on LncRNA P5848 (Figure 3E).

**Figure 3:** LncRNA P5848 induces ENO1 expression (**A**) Representative blots showing that LncRNA P5848 induces ENO1 expression after heat exposure, whereas knockdown of LncRNA P5848 suppresses ENO1 expression. (**B**) LncRNA P5848 promotes *ENO1* mRNA expression, while knockdown of LncRNA P5848 inhibits *ENO1* mRNA expression. (**C**) Schematic model for LncRNA P5848 regulating the expression of ENO1 and (**D**) luciferase assay showing LncRNA P5848 up-regulates *ENO1* mRNA. (**E**) Representative immune-fluorescent images for ENO1 showing the increase in ENO1 expression after heat exposure. *P<0.05, **P<0.01.

### Suppressing ENO1 counteracts the effect of LncRNA P5848

Since we have observed the up-regulating effect of LncRNA P5848 on ENO1 expression, we speculated that suppressing ENO1 would be able to counteract the effect of LncRNA P5848 on cell proliferation, apoptosis, and migration. Indeed, we found that knockdown of ENO1 significantly suppressed cell growth after heat exposure and co-suppressing ENO1 and LncRNA P5848 further inhibited cell growth Figure 4A. On the other hand, heat exposure at 50°C significantly decreased cell apoptosis, while knockdown of LncRNA P5848 markedly induced apoptotic cell death. Of note, knockdown of ENO1 further induced cell apoptosis in addition to LncRNA P5848 knockdown (Figure 4B). Also, knockdown of ENO1 could overcome the anti-apoptotic effect of LncRNA P5848 (Figure 4C), evident from the increase in expression level of pro-apoptotic protein BAX and activation of caspase-3 cleavage, while decreasing the level of anti-apoptotic protein Bcl-2. Co-suppressing ENO1 and LncRNA P5848 further enhanced the apoptotic effect (Figure 4C). Furthermore, knockdown of ENO1 suppressed the cell migration promoting effect of LncRNA P5848 (Figure 4D). Together, the data suggest that targetting LncRNA P5848 and ENO1 axis could inhibit tumor cells growth, survival, and migration.

**Figure 4:** Suppressing ENO1 counteracts the effect of LncRNA P5848 (**A**) Knockdown of ENO1 suppresses the cell growth promoting effect of LncRNA P5848. (**B**) Knockdown of LncRNA P5848 induces cell apoptosis and knockdown of ENO1 further enhances this effect. (**C**) Representative blots showing the expression level of BAX, Bcl-2, Cleaved caspase-3. β-actin functions as an internal loading control. ENO1 increases the expression level of anti-apoptotic protein Bcl-2 and reduces caspase-3 cleavage, while decreasing the level of pro-apoptotic protein BAX. (**D**) Knockdown of ENO1 or LncRNA P5848 suppresses the cell migration.

### LncRNA P5848 promotes tumor growth *in vivo*

We also examined the effect of LncRNA P5848 and ENO1 on tumor growth *in vivo*. Overexpression of LncRNA P5848 promoted tumor growth, while inhibiting LncRNA P5848 expression led to tumor regression as indicated by the tumor volume (Figure 5A,B). Besides, knockdown of ENO1 could counteract tumor growth induced by LncRNA P5848 (Figure 5A). Suppression of ENO1 further inhibited tumor growth in addition to the LncRNA P5848 knockdown (Figure 5C).

**Figure 5:** LncRNA P5848 promotes tumor growth *in vivo* Overexpression of LncRNA P5848 promotes tumor growth, while inhibiting LncRNA P5848 expression leading to tumor regression as indicated by the tumor volume (**A**), tumor weight (**B**). Suppression of ENO1 expression can further inhibit tumor in addition to the LncRNA P5848 knockdown (**C,D**). *P<0.05.

## Discussion

Here we have demonstrated a strong antitumor effect via targetting an LncRNA, P5848 *in vitro* and *in vivo*. We have verified the role of LncRNA P5848 in promoting cancer cell growth, invasion, and survival *in vitro* and *in vivo*; and have demonstrated that LncRNA P5848 is sufficient to drive cancer cell proliferation and migration, providing a possible explanation for the pro-metastatic properties of LncRNA P5848. Mechanistically, LncRNA P5848 functions through the up-regulation of ENO1 to bring about these effects.

A wealthy line of compelling evidence are indicating that LncRNAs have been substantially implicated in cancer development and progression [3,4], and with the findings from genome-wide cancer mutation analyses that show an extensive landscape of functional mutations within the noncoding genome, which impose substantial effects on the expression of LncRNAs [10,11]. While the exquisite regulation of LncRNA transcription can provide signals of malignant transformation, now with great advancements and efforts, it has been revealed that LncRNAs drive many clinically important cancer phenotypes through their interactions with other cellular macromolecules, which include DNA, protein, and RNA [11]. Recent advancements in dissecting the underlying mechanism for the roles of LncRNAs in cancer development and progression are offering great approaches to functionally annotate these cancer-associated transcripts, which in turn makes these molecules attractive therapeutic targets for intervention in the fight against cancer, such as HCC.

In the present study, we have also demonstrated that LncRNA P5848 can promote HCC cell growth, proliferation, invasion, migration, and survival *in vitro* and *in vivo.* We showed that LncRNA P5848-ENO1 axis contributes to HCC development and metastasis, as shown in our mouse model. Our studies suggest that therapeutic targetting strategies aimed at LncRNA P5848-ENO1 axis may have benefits for patients with HCC, especially given the role of EMT in metastasis, drug resistance, and poor prognosis.

The present study adds to a growing body of molecular evidence linking LncRNAs to cancer. For example, LncRNAs have been implicated in cell migration and invasion. Now in the present study, we add ENO1 as a downstream cellular target of LncRNA P58948 which can inhibit cell proliferation, invasion, and migration in HCC. However, additional signaling mechanisms involved in LncRNA P5848 driven cancer development and progression cannot be excluded.

In summary, we have demonstrated that ENO1 is a crucial downstream target of LncRNA P5848 to promote HCC cell growth, invasion, migration, and survival. The identification of LncRNA P5848-ENO1 axis could provide a new insight into the understanding on HCC initiation and progression, and it can bestow diagnostic and therapeutic advantages to the development of novel therapy of advanced HCC.

## Supplementary Material

Supplementary Table S1

## Abbreviations

Bax: BCL2-Associate
BCL2: B-cell lymphoma-2
DMEM: dulbecco’s modified eagle medium
EMT: epithelial to mesenchymal transition
ENO1: Enolase 1
GAPDH: glyceraldehyde-3-phosphate dehydrogenase
HCC: hepatocellular carcinoma
HRP: horse radish peroxidase
TBST: Tris Buffered Saline Tween
